The article "The Effect of miR-338-3p on HBx Deletion-Mutant (HBx-d382) Mediated Liver-Cell Proliferation through CyclinD1 Regulation" was retracted in 2013. Reasons: manipulated images; duplicated images; duplicated data.

# The Effect of miR-338-3p on HBx Deletion-Mutant (HBx-d382) Mediated Liver-Cell Proliferation through CyclinD1 Regulation

**DOI:** 10.1371/journal.pone.0043204

**Published:** 2012-08-17

**Authors:** Xiaoyu Fu, Deming Tan, Zhouhua Hou, Zhiliang Hu, Guozhen Liu, Yi Ouyang, Fei Liu

**Affiliations:** 1 Department of Infectious Disease, Xiangya Hospital, Central South University, Changsha, Hunan, China; 2 The Second Hospital of Nanjing, Nanjing, Jiangsu, China; Inserm, U1052, UMR 5286, France

## Abstract

**Objective:**

Hepatitis B Virus (HBV) DNA integration and HBV X (HBx) deletion mutation occurs in HBV-positive liver cancer patients, and C-terminal deletion in HBx gene mutants are highly associated with hepatocarcinogenesis. Our previous study found that the HBx*-*d382 deletion mutant (deleted at nt 382–400) can down-regulate miR-338-3p expression in HBx-expressing cells. The aim of the present study is to examine the role of miR-338-3p in the HBx-d382-mediated liver-cell proliferation.

**Methods:**

We established HBx-expressing LO2 cells by Lipofectamine 2000 transfection. A miR-338-3p mimics or inhibitor was transfected into LO2/HBx-d382 and LO2/HBx cells using miR-NC as a control miRNA. *In silico* analysis of potential miR-338-3p targets revealed that miR-338-3p could target the cell cycle regulatory protein CyclinD1. To confirm that CyclinD1 is negatively regulated by miR-338-3p, we constructed luciferase reporters with wild-type and mutated CyclinD1-3′UTR target sites for miR-338-3p binding. We examined the CyclinD1 expression by real-time PCR and western blot, and proliferation activity by flow cytometric cell cycle analysis, Edu incorporation, and soft agar colony.

**Results:**

HBx-d382 exhibited enhanced proliferation and CyclinD1 expression in LO2 cells. miR-338-3p expression inhibited cell proliferation in LO2/HBx-d382 cells (and LO2/HBx cells), and also negatively regulated CyclinD1 protein expression. Of the two putative miR-338-3p binding sites in the CyclinD1-3′UTR region, the effect of miR-338-3p on the second binding site (nt 2397–2403) was required for the inhibition.

**Conclusion:**

miR-338-3p can directly regulate CyclinD1 expression through binding to the CyclinD1-3′UTR region, mainly at nt 2397–2403. Down-regulation of miR-338-3p expression is required for liver cell proliferation in both LO2/HBx and LO2/HBx-d382 mutant cells, although the effect is more pronounced in LO2/HBx-d382 cells. Our study elucidated a novel mechanism, from a new miRNA-regulation perspective, underlying the propensity of HBx deletion mutants to induce hepatocarcinogenesis at a faster rate than HBx.

## Introduction

Among the four open reading frames (ORFs) in the genome of hepatitis B virus (HBV), the HBV X gene (HBx) correlates the most to liver cancer development like hepatocellular carcinoma (HCC). The HBx protein is a multifunctional regulator that is essential for viral replication and plays an important role in regulating gene transcription, participating in cell signaling, and controlling cell proliferation and apoptosis [1]–[2]. However, there is controversy surrounding the direct causal effect of HBx on HCC development [3]–[5]. The integration of the HBx gene into the host genome in hepatocarcinoma tissues, and the gene mutants in HBx that arise due to this integration process, have been reported in many studies. The study conducted by Minenura M et al. [6] revealed a correlative relationship between HBx gene point mutations (at codon 130 [AAG → ATG] and 131 [GTC → ATC]) and liver cancer. Another report by Yeh et al. [7] found that HBx*-*A31 (containing a mutation at codon 31) was detected more frequently in patients with HCC. Constructs based on either naturally occurring or artificially designed carboxyl-terminal HBx gene deletion mutants were successfully cloned and encoded a carboxy-terminal truncated HBx protein. These HBx mutants have very different functions than wild-type HBx protein [8]–[9], since the mutants exhibited the ability to promote cell proliferation and to reduce the response to apoptotic stimuli [9]–[10] that play important roles in HCC development. However, the mechanism underlying HBx deletion mutant-induced malignant transformation of liver cells is still unclear.

MicroRNAs (miRNAs) are a class of endogenous, noncoding small RNAs that regulate gene expression at the post-transcriptional level through binding the 3′-UTR region of the target gene mRNA. Several recent studies have shown that dysregulation of miRNA expression is associated with a variety of tumors, and that these miRNAs may play a tumor suppressor or oncogenic role [11]–[12]. Important to our present study, miRNAs have been reported to be closely related to the incidence and development of liver cancer [13]–[15]. However, only a few studies have evaluated the specific roles of either the HBx deletion mutants or miRNAs, or their possible interaction, in the incidence and development of HBV-related liver cancer.

Our previous studies found that liver cancer tissues from chronically HBV-infected human patients contained an elevated incidence of a particular HBx deletion mutation, HBx-d382 (named because of a deletion mutation between nt 382–400) [16]. We speculated that this relationship was related to the higher incidence of HBx mutations that occur following HBV DNA integration, which often happens during chronic HBV infection that also correlates with the development of hepatocarcinoma. Upon further investigation by miRNA microarray analysis, we found that stable expression of HBX or HBx-d382 in LO2 cells decreased miRNA expression, including miR-338-3p, as compared to control LO2/pcDNA cells; interestingly, the LO2/HBx-d382 cells exhibited this phenotype in a more pronounced way than LO2/HBx cells. Additional analysis by real-time PCR confirmed this result (unpublished data). Furthermore, the miRNA target prediction based on bioinformatic analysis showed that CyclinD1 is a likely miR-338-3p target. To better understand the influence of the down-regulated miR-338-3p expression in cells expressing the HBx-d382 mutant and to determine whether there are any changes in miR-338-3p-mediated CyclinD1 expression, we used the stably transfected LO2/HBx and LO2/HBx-d382 (also used in our previously published experiments) as our experimental model. The results of our study suggest that the miR-338-3p-mediated CyclinD1 expression changes downstream of HBx mutant gene function may help to understand the mechanisms underlying the HBx-d382 mutant-induced hepatocarcinogenesis from a new perspective.

## Materials and Methods

### Cells Culture and Establishment of the Stably Transfected Cell Lines

All cells were cultured in RPMI-1640 medium (GIBCO, USA) containing 10% fetal bovine serum (FBS) (GIBCO, USA) and 100 units/mL penicillin plus 100 µg/mL streptomycin at 37°C with 5% CO2. The control plasmid pcDNA3.0, recombinant plasmid pcDNA3.0/HBx-d382 (a mutant of the HBx gene with deletion from 382–400 bp), and pcDNA/HBx were previously established in our lab [16]. The HBx genetic fragments used here originate from the liver cell line HepG2.215. We established stably engineered LO2 cells transfected with the wild type HBx and HBx-d382 mutant plasmids; the hepatocyte cell line LO2 (obtained from Chinese Academy of Science, Cell Biology of Shanghai Institute) was transfected with Lipofectamine^TM^2000 (Invitrogen, California, USA) according to the manufacturer’s instructions and was selected with G418 (Geneticin, GIBCO, USA). Empty pcDNA3.0 vector plasmid was used as a control. The stable transfection of pcDNA3.0/HBx-d382 (termed LO2/HBx-d382), pcDNA/HBx (termed LO2/HBx), or the empty vector (termed LO2/pcDNA3.0) was confirmed by RT-PCR for gene expression and western blotting for protein expression.

**Figure 1:** HBx-d382 enhances the non-anchored growing ability of transfected hepatocytes. (A–B) The identification of stable HBx transfection in LO2 cells. (A) The HBx gene was identified by RT-PCR. (B) Western blotting showed the expression of HBx in LO2 cells. 1: LO2; 2: LO2/pcDNA3.0; 3: LO2/HBx-d382; 4: LO2/HBx; M: marker. (C) Soft agar colony formation assay of transfected LO2 cells. The rate of colony formation in HBx-expressing cells was significantly higher than in control LO2 and LO2/pcDNA3.0 cells (*P<0.01). While within the groups of LO2/HBx-d382 LO2/HBx, the former was higher than the latter (#*P*<0.01).

### Cell Transfection

HBx-expressing cells were transfected with miRNA mimics or miRNA inhibitor (GeneCopoeia, USA) using Lipofectamine 2000 (Invitrogen) at a final concentration of 50 nM, according to manufacturer’s instructions. The normal recommended controls for the miRNA-mimics and inhibitor (GeneCopoeia, USA) were used in the experiments. Changes in gene expression were detected 48 hr after transfection. miR-338-3p miRNA target verification was performed in LO2/HBx cells, which were co-transfected with miR-338-3p mimics and the dual luciferase reporter plasmid. miRNA-NC miRNA was used as the control for miR-338-3p.

### Inhibition of HBx Expression

Small interfering RNA (siRNA) sequences specifically targeting HBx were selected accordingly [17] and synthesised by GenePharma (Shanghai, China). Approximately 50 nM HBx siRNA or control siRNA was transfected into LO2/HBx and LO2/HBx-d382 cells by Lipofectamine as described above.

**Figure 2:** HBx, especially HBx-d382, enhances CyclinD1 expression. (A) CyclinD1 protein level of the engineered LO2 cells. (B) The histogram of CyclinD1 mRNA and protein level in LO2/HBx and LO2/HBx-d382 cells, compared with LO2/pcDNA3.0 cells (*P<0.001,**P = 0.017,***P = 0.029).

### RT-PCR Analysis

Total RNA from the engineered LO2 cells was extracted by Trizol (Invitrogen, USA). The PCR primers used for HBx detection were as follows: for HBx, 5′-AAGGTACCATGGCTGCTAGGCTGTGCT-3′ (forward) and 5′-CTGGGCCCTTAGGCAGAGGTGAAAAAGTTG-3′ (reverse), leading to a 462 bp amplified product; for the β-actin control, 5′-CTCCATCCTGGCCTCGCTGT-3′ (forward) and 5′-GCTGTCACCTTCACCGTTCC-3′ (fragment), leading to a 242 bp amplified product.

### Soft Agar Colony Formation Assay

The assay was conducted according to previously published methods [18], with slight modifications. Briefly, 5×10^3^ transfected LO2 cells were first thoroughly mixed with 2 mL RPMI Medium 1640 containing 3 g/L agar and 10% FBS. This mixture was then added onto solid agar (RPMI Medium 1640 medium containing 5 g/L agar and 10% FBS) in a 6-well plate and incubated for 2 weeks. Finally, the derived clones from each group within a randomly selected area were selected and counted under a microscope at 50× magnification.

### Quantitative Real-time PCR (qRT-PCR) Analysis

miR-338-3p expression in normal hepatocytes (LO2 and QSG7701 cells) and HBx-expressing cells after knocking down HBx expression was measured with SYBR qRT-PCR. CyclinD1 expression before and after miR-338-3p mimic or inhibitor introduction into HBx-expressing LO2 cells was measured with SYBR qRT-PCR. Total RNA was extracted with Trizol (Invitrogen) according to the manufacturer’s instructions.

miR-388-3p cDNA was synthesized from 2 µg of total RNA with an All-in-one™ miRNA First-Strand cDNA Synthesis (GeneCopoeia) Kit using the supplied poly-A primer. Real-time PCR was performed in a 20 µL reaction mix including 2 µL of 5× diluted reverse transcription product, 2 µL miRNA specific primer, 10 µL SYBR 2× All-in-one qPCR Mix, 0.4 µL 50× ROX Reference dye, and 3.6 µL double distilled water. The cycling conditions for amplification on the 7500 Real-Time PCR System (Applied Biosystems, Foster City, CA) were 95°C for 10 min, followed by 40 cycles of 95°C for 10 sec, 60°C for 20 sec, and 72°C for 32 sec. The data were normalized against the U6 snRNA.

CyclinD1 expression was analyzed with THUNDERBIRD SYBR qPCR Mix (ToYoBo, Japan). cDNA was synthesized with the RevertAid™ First Strand cDNA Synthesis Kit (MBI Fermentas, Canada) in a total volume of 20 µL. The primer sequences used were as follows: for CyclinD1, 5′-AGGAACAGAAGTGCGAGGAGG-3′ (forward) and 5′-GGATGGAGTTGTCGGTGTAGATG-3′ (reverse); for GAPDH, 5′-CGGATTTGGTCGTATTGGGC-3′ (forward) and 5′-CCTGGAAGATGGTGATGG.

GATT-3′ (reverse). qRT-PCR was performed on an Applied Biosystems 7500 RT-PCR System. The cycling conditions for amplification were as follows: 95°C for 1 min, 40 cycles of 95°C for 15 sec, and 58°C for 35 sec. The data were normalized against GAPDH. Each sample was analyzed in triplicate, and the fluorescence signal was measured at each extension step. The relative expression was determined using the 2^−ΔΔCT^ method, where the normalized CT (ΔCT) value was calculated by subtracting the CT of a control gene (U6 snRNA for miR-338-3p and GAPDH for CyclinD1) from the CT of the gene of interest.

**Figure 3:** miR-338-3p inhibits cell proliferation, especially in LO2/HBx-d382 cells. (A) A representative cell cycle profile for miR-338-3p mimics or inhibitor in LO2/HBx-d382 and LO2/HBx cells comparing to their control RNA transfection. (B) Average of G1 phase populations in HBx-expressed LO2 cells after transfected miR-338-3p mimics or inhibitor (*P<0.001). (C) Average of S phase populations after transfected miR-338-3p mimics or inhibitor in LO2/HBx-d382 and LO2/HBx cells (*P<0.001). While miR-338-3p overexpresses or suppresses, miR-338-3p induce cell cycle arrest and anti-miR-338-3p increases cell growth, especially in LO2/HBx-d382 cells. Values in (B) and (C) are means ±SD of three separate experiments.

**Figure 4:** miR-338-3p inhibits cell proliferation by Edu assay. (A–B) Representative profiles of Edu cell proliferation after transfection with miR-338-3p mimics or inhibitor in LO2/HBx-d382 and LO2/HBx cells compared to their negative control transfection (magnification 100×). (C) Rate of Edu positive cells in S phase. Gain of miR-338-3p inhibits the cellular DNA replication in HBx-expressed LO2 cells and control cells, whereas loss of miR-338-3p expression demonstrates an adverse result, especially in LO2/HBx-d382 cells. (*P<0.001; **P<0.01; ***P<0.05).

**Figure 5:** miR-338-3p influence the colony formation of transfected LO2 cells. (A–B) Gain of miR-338-3p decreases the rate of colony formation of LO2/HBx-d382 and LO2/HBx cells, whereas loss of miR-338-3p enhances the non-anchored growing ability in HBx-expressing cells (*P<0.001, **P<0.01). (C) The non-anchored growing ability of control LO2/pcDNA3.0 cells are also inhibited by miR-338-3p, although the significant difference is lower than that in HBx-expressing cells (***P = 0.032,#*P* = 0.025).

### Western Blot Analysis

HBx and CyclinD1 proteins were measured by western blot. Total protein was extracted from transfected cells using the RIPA lysis buffer (Beyotime, China) according to the manufacturer’s instructions. For western blot analysis, equal amounts of protein samples were separated by 10% SDS-PAGE and transferred onto PVDF membranes (Millipore, USA). Blots were blocked using with 5% skim milk, followed by incubation with antibodies specific for rabbit anti-HBx (Abcam, England, 1∶1500 dilution) or mouse anti-CyclinD1 (Santa Cruz, USA, 1∶100 dilution), and mouse anti-β-actin (Abcam, 1∶3000 dilution). Blots were then incubated with goat anti-rabbit or anti-mouse secondary antibody conjugated to horseradish peroxidase (Jackson Immunoresearch, USA, 1∶5000 dilution) and visualized by enhanced chemiluminescence (ECL) (Amersham Biosciences, USA).

### Gene Sequence Analysis and Primer Design

Through *in silico* miRNA target prediction, we found two binding sites for miR-338-3p in the 3′ untranslated regions (3′-UTR) of CyclinD1. Two gene fragments corresponding to the two binding sites in CyclinD1-3′-UTR were cloned into a vector using the restriction enzymes XhoI and NotI. Using the NM_053056 (gene = “CCND1”) gene sequence, primers were designed to amplify binding site locations in the 3′-UTR region. Mutation primers mutating the specific binding sequence for miR-338-3p in CyclinD1 were also designed, named Mut (mutating both binding sites), Mut-1 (mutating nt 907–913), or Mut-2 (mutated nt 2397–2403). The PCR products were cloned into a pmirGLO Vector (Promega, Madison, WI, USA) that was designed to quantitatively evaluate miRNA binding and function by measuring luciferase activity after inserting miRNA target sites downstream or 3′ of the luciferase gene. In this vector, Renilla luciferase was used as the primary reporter, while firefly luciferase acts as a control reporter for normalization and selection. PCR products were 1573 bp in size.

The primers used for cloning were as follows: **Wt**-Forward: 5′- CCGCTCGAGTC CTATTTTTGTAGTGACCTGTTTATG-3′, **Wt**-Reverse: 5′- GAATGCGGCCGCGC TA CGCCCCCGATCAGATGAAG-3′; **Mutant**-Forward: 5′-CCGCTCGAGTCC TAT TTTTGTAGTGACCTGTTTATGAG***TTCCAGA***TTTTCTACCCAACGGCCC-3′, **Mutant**-Reverse: 5′-GAATGCGGCCGCGCTACGCCCCCGATCAGATGAAGT.

GC***TCTGGAA***CACAGGCGCAGGGAAGAGAAG-3′; **Mutant1**-Forward: 5′-CCGC

TCGAGTCCTATTTTTGTAGTGACCTGTTTATGAG***TTCCAGA***TTTTCTACCCAACGGCCC-3′, **Mutant1**-Reverse: 5′-GAATGCGGCCGCGCTACGCCCCCGATCAGAT

GAAG-3′; **Mutant2**-Forward: 5′-CCGCTCGAGTCCTATTTTTGTAGTGACCTGT

TTATG-3′, **Mutant2**-Reverse: 5′-GAATGCGGCCGCGCTACGCCCCCGATCAGATG

AAGTGC***TCTGGAA***CACAGGCGCAGGGAAGAGAAG-3′.

**Figure 6:** CyclinD1 is a direct target of and is regulated by miR-338-3p, and the effect of miR-338-3p on CyclinD1 is mainly dependent on the CyclinD1-3′-UTR region (nt 2397–2403). (A–B) Successfully constructed plasmids of CyclinD1-3′-UTR. (A) Amplification of a DNA fragment containing CyclinD1-3′-UTR region. PCR amplification was performed using specific primers for the types of WT-, Mut-, Mut1-, and Mut2-Cyclin D1-3′-UTR, respectively, and genomic DNA isolated from the genome of LO2/HBx cells was used as PCR template. An approximately 1573 bp band PCR product was detected by agarose gel electrophoresis. (B) Identification of recombinant plasmids. The fragment digested with XhoI and NotI from the recombinant plasmids: pCyclinD1-3′-UTR-WT, pCyclinD1-3′-UTR-Mut, pCyclinD1-3′-UTR-Mut1, and pCyclinD1-3′-UTR-Mut2 were used as a template for confirmation PCR. The PCR product was about 1573 bp, which was finally confirmed by DNA sequencing. miR-338-3p targets CyclinD1. (C) Dual luciferase assay of LO2/HBx cells cotransfected with the Renilla luciferase constructs containing the CyclinD1 WT or Mut 3′-UTR and miR-338-3p mimics or negative RNA (*P = 0.404,**P<0.001). (D) The major site of CyclinD1 targeted by miR-338-3p was at position 2397–2403 nt. Effects of miR-338-3p and the negative control on the reporter constructs containing CyclinD1-3′-UTR Mut1 and Mut2 were determined 48 hours after transfection. Renilla luciferase values normalized to Firefly luciferase are presented. (**P<0.001,***P = 0.04). (E–G) CyclinD1 protein expression after transfection of miR-338-3p mimics, inhibitor, or negative control (*P<0.001,**P<0.01). The fold change before and after transfection is more pronounced in LO2/HBx-d382 cells than that in LO2/HBx and control cells. Data are shown as mean ±SD from at least 3 independent experiments. (H) qRT-PCR with the 2^−ΔΔCT^ method to evaluate the CyclinD1 mRNA expression normalized to GAPDH in LO2/HBx-d382, LO2/HBx, and control cells transfected with miR-338-3p mimics or inhibitor or their respective controls(★*P* = 0.164,★★ *P* = 0.438, #*P* = 0.220,##*P* = 0.101,* *P* = 0.254,** *P* = 0.417).

### Amplification and Identification of CyclinD1-3′-UTR Constructs

Amplification of wild-type and mutant plasmids was carried out using the same conditions. Briefly, 6 µL of 5× PrimeSTAR buffer (TaKaRa, Japan), 2 µL of 2.5 mM dNTPmix, 1 µL each of upstream and downstream primer (10 mM), 0.3 µL of PrimeSTAR HS DNA polymerase (2.5 U/µL), 1 µL of DNA template, and sterile water up to a total of 30 µL per reaction were mixed together. Touchdown PCR was used for amplification as follows: hot-start at 95°C for 5 min, followed by 10 cycles of denaturation at 98°C for 10 sec, annealing starting from 65°C and decreasing 1°C in each cycle, and extension at 72°C for 1 min 45 sec; for the remaining 18 cycles, the annealing temperature was kept at 55°C. A final extension step at 72°C for 7 min followed by decreasing the temperature to 4°C completed the PCR reaction. To verify the PCR products, 2 µL of DNA sample was loaded on 1% agarose for gel electrophoresis. PCR products were retrieved from the gel and double digested with XhoI and NotI. Meanwhile, double digestion of pmirGLO vectors with XhoI and NotI had been performed. The digested fragments from the vector and PCR products were purified and used to clone recombinant plasmids, including wt/Mut-CyclinD1-3′-UTR, CyclinD1-3′UTR-Mut1, and CyclinD1-3′UTR-Mut2. To identify the recombinant plasmids, the inserts were double digested with XhoI and NotI.

### Identification of miR-338-3p Target by Dual-luciferase Reporter Assay

The reporter assay was performed according to Promega's instructions. Briefly, growth medium was removed from cultured cells, fresh medium (100 µL/well) was added, and luciferase substrate (100 µL/well) was prepared. The plate was gently rocked at room temperature for 10 min, and firefly luciferase activity (hLuc) was then measured using a microplate luminometer (Veritas™ microplate fluorescence reader; YuanPingHao Bio, Beijing, China). Next, 100 µL of Stop & Glo reagent was dispensed, incubated for 10 min by gentle rocking, and Renilla luciferase activity (hRluc) was measured. The luciferase counts were then normalized to hLuc counts to obtain final reporter activity. Each sample was measured in triplicate.

### EdU Assay

Cell proliferation was measured by 5-ethynyl-2′-deoxyuridine (EdU) assay using an EdU assay kit (Ribobio, Guangzhou, China) according to the manufacturer’s instructions. Brieﬂy, LO2/HBx-d382 and LO2/HBx cells were cultured in triplicate at 5×10^3^ cells per well in 96-well plates and were transfected with 50 nM of miR-338-3p mimics, miR-338-3p inhibitor, or their respective control RNA for 48 h. The cells were then exposed to 50 µM of EdU for additional 4 h at 37°C. The cells were then fixed with 4% formaldehyde for 15 min at room temperature and treated with 0.5% Triton X-100 for 20 min at room temperature for permeabilization. After 3× washes with PBS, the cells were treated with 100 µL of 1× Apollo^R^ reaction cocktail for 30 min. Subsequently, the DNA contents of each well of cells were stained with 100 µL of Hoechst 33342 (5 µg/mL) for 30 min and visualized under a ﬂuorescent microscope (Olympus, Japan).

### Cell Cycle Assay

Cell cycle analysis was determined by flow cytometry (BD, UA). Brieﬂy, LO2/HBx-d382 and LO2/HBx cells at 1×10^6^ cells per well were cultured in 6-well plates and transfected with 50 nM of miR-338-3p mimics, miR-338-3p inhibitor, or their respective control RNA for 48 h. The cells were then harvested and fixed in 70% ice-cold ethanol for 24 h, followed by propidium iodide (PI) staining. The different cell cycle phases were analyzed using a FACS Calibur instrument.

### Statistical Analysis

The data from soft agar colony formation and CyclinD1 expression in the engineered LO2 cells was performed with Fisher’s Least Significant Difference (LSD)-*t* test. The data from miR-338-3p expression in normal hepatocytes was performed with Fisher’s Least Significant Difference (LSD)-*t* test. All the other data was analyzed by unpaired two-tailed *t*-test. All data was expressed as means and standard deviation from at least 3 independent experiments. All *p* values were obtained with SPSS 16.0 software package, and a *p*<0.05 was considered statistically significant.

## Results

### HBx-d382 Enhances the Non-anchored Growing Ability of Transfected Hepatocytes and Promotes CyclinD1 Expression

There is an established correlation between the presence of HBx deletion mutations in liver cells and hepatocarcinogenesis. To study whether and how the HBx deletion mutation affected the growth and proliferation of hepatocytes, we observed the isolated effect of the HBx-d382 HBx deletion mutant, found previously in our studies to be prevalent in HCC patient tumors, on hepatocyte cell proliferation as compared to the wild-type HBx gene. To do this, we established a non-tumorigenic human hepatocyte cell line, LO2, expressing the mutated HBx-d382 gene as well as a control LO2 cell line expressing the wild-type HBx. We first used RT-PCR to identify the HBx gene in the cDNA of the engineered LO2 cells. β-actin was used as a loading control (Fig. 1A). The data showed that the HBx gene had been successfully introduced into the host genome in LO2 cells. Western blotting showed that HBx protein expression could be detected in LO2 cells (Fig. 1B). These data suggest that stably HBx-transfected LO2 cells were successfully established.

We used these engineered cells to test whether HBx-d382 had an effect on cell proliferation. Soft agar colony formation analysis revealed that the rate of colony formation in LO2/HBx-d382 and LO2/HBx groups was significantly higher than that of the control LO2 group and LO2/pcDNA3.0 groups after culturing for 2 weeks (*p*<0.01); there was no significant difference in colony formation between the control LO2 and LO2/pcDNA3.0 groups (Fig. 1C). Within the LO2/HBx-d382 and LO2/HBx groups, the former was higher than the latter (*p*<0.01). This result indicated that HBx and HBx-d382 led to cell cycle dysregulation, with the HBx-d382 mutant leading to the most pronounced proliferation effect. As the cyclin proteins are known to regulate cell proliferation and cell cycle, we tested whether CyclinD1 was differentially expressed in the engineered LO2 cells. PCR and western blot results showed that CyclinD1 mRNA and protein levels, respectively, were up-regulated in cells transfected with HBx and HBx-d382, when compared with those transfected with pcDNA3.0 (Fig. 2); consistent with the data in Figure 1, the effect of HBx-d382 on CyclinD1 expression was more prominent than wild-type HBx. This result indicated that HBx and the HBx-d382 deletion mutant increased CyclinD1 expression in hepatocytes.

### Relative Expression of miR-338-3p in Normal Hepatocytes is Higher than that in HBx-expressing Cells

Our unpublished studies showed that miR-338-3p was down-regulated in HBx-expressing LO2 cells compared with control LO2/pcDNA3.0 cells by microarray and real-time PCR; however, whether miR-338-3p expression was altered in normal hepatocytes compared to HBx-expressing cells was unknown. To address this, real-time PCR evaluation using the 2^−ΔΔCT^ method showed that the relative expression of miR-338-3p in normal hepatocytes is higher than that in HBx-expressing cells (Fig. S1). Moreover, according to the results from Figure 2, we conclude that CyclinD1 expression inversely correlates with miR-338-3p expression in HBx-expressing LO2 cells.

### miR-338-3p Inhibits Cell Proliferation, Especially in LO2/HBx-d382 Cells

We next wanted to determine whether the HBx-regulated miRNA miR-338-3p that we identified in our miRNA microarray could regulate the HBx-mediated increased proliferation we observed in Figure 1. To examine the functional role of miR-338-3p, we altered cellular miR-338-3p expression by transfecting the HBx- and HBx-d382–expressing LO2 cells with miR-338-3p mimics or an miR-338-3p inhibitor compared with LO2/pcDNA3.0 cells. Cell cycle and EdU incorporation assays were used to determine cell proliferation. Compared to their respective negative controls (NC), the HBx-expressing LO2 cells transfected with the miR-338-3p mimics displayed significantly higher frequency of cells at the G1 phase and a lower frequency of cells at S phase (Fig. 3A–C, Fig. S2, *p*<0.001). In contrast, cells transfected with miR-338-3p inhibitor showed a significant decrease of cells at G1 phase and an increase of cells at S phase (Fig. 3A–C, Fig. S2, *p*<0.001). This indicated that miR-338-3p inhibited cell cycle progression from the G1 phase to the S phase. Next, we used the EdU incorporation assay, which is a more sensitive and specific method [19]–[20], to evaluate the effects of miR-338-3p on cell proliferation. We found that the number of cells incorporating EdU in the miR-338-3p mimic-treated group was significantly reduced as compared to the negative control. In contrast, the number of cells incorporating EdU was significantly increased in the miR-338-3p inhibitor-treated group as compared with the negative control. Interestingly, this effect is especially significant in LO2/HBx-d382 cells (Fig. 4A–C). In addition to regulating cell cycle transition between the G1/S phase, this result indicated that miR-338-3p also inhibited cell proliferation, especially in LO2/HBx-d382 cells. Finally, the effects of miR-338-3p mimics/inhibitors on the colony-forming assay demonstrated that the miR-338-3p inhibited the non-anchored growing ability of transfected LO2 cells, especially in HBx-expressing cells (Fig. 5).

### CyclinD1 is a Direct Target of miR-338-3p, and the Effect of miR-338-3p on CyclinD1 is Mainly Dependent on the CyclinD1-3′-UTR Region (nt 2397–2403)

As predicted by several *in silico* methods for target-gene prediction, including TargetScan [21], CyclinD1 was identified as one of the candidate genes regulated by miR-338-3p. Two putative binding sites, nt 907–913 and nt 2397–2403, are located in the CyclinD1-3′-UTR. To determine which putative binding site is used by miR-338-3p, or whether both are used, we mutated each of these putative sites alone (Mut1-CyclinD1-3′-UTR [mutated nt 907–913] and Mut2-CyclinD1-3′-UTR [mutated nt 2397–2403nt]) as well as both of these sites together (Mut-CyclinD1-3′-UTR) in the 3′-UTR region of the CyclinD1 gene. WT-CyclinD1-3′-UTR was used as a control. PCR amplification was performed using specific primers for the mutated binding sites. The amplified PCR products and genomic DNA isolated from the genome of LO2/HBx cells was used as a PCR template. As shown in Figure 6A, the different CyclinD1-3′-UTR gene-derived PCR products were found around the predicted 1573 bp band size. The plasmids were then extracted and subjected to a double digestion with XhoI and NotI enzymes that generated one product: a band at approximately 1573 bp (Fig. 6B) that corresponds to the CyclinD1-3′-UTR gene for all plasmids. Finally, the recombinant plasmid gene sequences were further verified by DNA sequencing.

To validate whether miR-338-3p can directly regulate CyclinD1 through either or both of the putative binding sites in the 3′-UTR region of CyclinD1, the WT-, Mut-, Mut1-, and Mut2-CyclinD1-3′-UTR plasmids were cloned into the 3′-UTR of the Renilla luciferase gene and were co-transfected with miR-338-3p mimics or negative control RNA in LO2/HBx cells. The luciferase enzyme activity levels were then measured to determine the miR-338-3p effects on luciferase translation upon binding to the WT or mutated 3′-UTR regions from CyclinD1. Compared with the negative control group, Renilla luciferase activity was significantly decreased (i.e. the ratio of hRluc to hLuc deceased) in the group co-transfected with miR-338-3p and pCyclinD1-3′-UTR-WT (Fig. 6C, *p*<0.001), as predicted. However, luciferase activity in the group co-transfected with miR-338-3p and pCyclinD1-3′-UTR-Mut did not exhibit a significant difference from the NC group (*p* = 0.404), indicating that miR-338-3p could no longer bind. To determine if one or both of the binding sites were necessary for the functional effect of miR-338-3p, we compared the luciferase activity between pCyclinD1-3′-UTR-Mut1 and pCyclinD1-3′-UTR-Mut2 groups with the negative control group. The CyclinD1-3′-UTR-Mut1 maintained the significant difference (*p*<0.001) noted in the pCyclinD1-3′-UTR-WT in response to miR-338-3p as compared with the negative control group, indicating that miR-338-3p was independent of this binding site. In contrast, the luciferase activity in pCyclinD1-3′-UTR-Mut2 group was less affected by miR-338-3p (Fig. 6D, *p* = 0.04), indicating that this binding site is important for miR-338-3p binding and function. These data indicated that miR-338-3p has effect on both binding sites in CyclinD1-3′-UTR region, but that the main binding site is the second site (nt 2397–2403).

### miR-338-3p Represses CyclinD1 Protein Expression

To directly test the validity of the putative target, HBx-expressing LO2 cells were transfected with miR-338-3p mimics or miR-338-3p inhibitor as well their respective negative controls. The mRNA and protein levels of CyclinD1 were measured by qRT-PCR and Western blotting, respectively. Relative to the control, miR-338-3p overexpression downregulated endogenous CyclinD1 protein, while miR-338-3p inhibition upregulated the CyclinD1 protein; consistent with our previous data, these changes in CyclinD1 are more prominent in the LO2/HBx-d382 cells (Fig. 6E–G). In contrast, no change of CyclinD1 mRNA level was noted (Fig. 6H), indicating post-transcriptional regulation of CyclinD1 by miR-338-3p.

### Changes in HBx Expression Affect miR-338-3p and CyclinD1 Expression in Transfected LO2 Cells

Since the miR-338-3p and CyclinD1 expression was significantly changed in HBx-expressing LO2 cells, we wondered whether the reduction of HBx could also lead to differential miR-338-3p and CyclinD1 expression. To address this question, we transfected HBx siRNA or control RNA into LO2/HBx and LO2/HBx-d382 cells to inhibit HBx expression. We measured the miR-338-3p expression by qRT-PCR using the 2^−ΔΔCT^ method 48 h after transfection and found that there was a significant increase of miR-338-3p expression after knocking-down HBx compared to the negative controls (Fig. S3), while the western blot showed that CyclinD1 protein levels were significantly down-regulated after HBx reduction (Fig. S3), Our findings revealed that high HBx expression up-regulated CyclinD1 and down-regulated miR-338-3p, while HBx reduction leads to down-regulated CyclinD1 and up-regulated miR-338-3p expression,indicating that HBx is necessary for cyclinD1 upregulation. Our data introduces a new mechanism suggesting that HBx up-regulated CyclinD1 through down-regulating miR-338-3p.

## Discussion

Although the integration of HBV DNA into the host genome is not required for viral replication, it is a common phenomenon that HBV genes integrate with host genomic DNA in many liver tissues chronically infected with HBV. This promotes HBV persistent infection [22]–[23] by providing protection of the viral genome from immunological surveillance and, most importantly, promoting the development of genomic DNA instability that contributes to malignant transformation of liver cells [24]–[25]. In addition to effecting these changes on the infected host liver cells, the process of HBV DNA integration can induce mutations in the HBV DNA itself. Deletion mutations are frequently found in the integrated HBV DNA, especially in the X gene (including the HBx gene explored here), S gene, and enhancer regions, resulting in the expression of truncated proteins encoded by the mutated genes, such as the truncated HBx protein that can then lead to dysregulation of host cellular genes [9], [26]. For the HBx gene, deletions in the C-terminal region of the gene are common after HBV DNA integration. In the context of hepatocarcinogenesis, there is an intriguing correlation between the occurrence of this particular mutation and transformed liver cancer cells, as the level of C-terminal truncated HBx protein is higher in transformed tumor tissues as compared to distal non-tumor tissues in HBV-infected HCC patients [10], [26]. Supporting this finding, Iavarone et al. [9] found that a truncated HBx protein detected in HCC tissues derived from an HBx gene deletion that led to a reading frame shift mutation and the emergence of a new STOP codon.

Currently, the mechanisms underlying how HBx induces hepatocarcinogenesis are not fully clear. Wang et al. [27] reported that HBx-mediated down-regulation of let-7a expression inhibited cell proliferation; this was the first study to report an interaction between HBx and miRNA. However, the role of miRNA in the relationship between the HBx deletion mutation and hepatocarcinogeness is largely unexplored. To better understand the mechanism underlying the effect of miRNAs on HBx deletion-mutation–related HCC, we performed the study described here, and our results provide new ideas for the diagnosis and treatment of liver cancer. Our previous studies found that the HBx-d382 mutant was detected in several HCC patients [16], and the ability of HBx-d382 to induce tumor formation was confirmed in a nude mice model [28]. miRNA microarray analysis and confirmatory real-time PCR data showed that HBx-d382 had a stronger ability to down-regulate miR-338-3p expression than wild-type HBx in transfected LO2 hepatocyte cells (unpublished data). To understand what genes targeted by miR-338-3p might function to promote HBx deletion-mutation related liver cancer, we used TargetScan to identify the potential miR-338-3p target gene and found that CyclinD1 was a likely candidate. Furthermore, HBx-d382 was able to promote proliferation and anchor-independent growth of LO2 cells as well as enhance CyclinD1 gene expression. Edu incorporation and cell cycle analysis by flow cytometry to measure cell proliferation demonstrated that ectopic expression of miR-338-3p mimics in both LO2/HBx and LO2/HBx-d382 cells inhibited cell proliferation, whereas repression of endogenous miR-338-3p expression enhanced cell proliferation. Furthermore, the forced expression or down-regulation of miR-338-3p reduced or enhanced, respectively, the protein expression of CyclinD1 in both LO2/HBx and LO2/HBx-d382 cells. In the above experiments, the phenotypes were more profound in LO2/HBx-d382 than in LO2/HBx cells. The dual luciferase reporter assay confirmed that CyclinD1 is a direct target gene of miR-338-3p, and that the main binding site of miR-338-3p in CyclinD1-3′-UTR region is located between nt 2397–2403 (the second predicted binding site). Finally, HBx reduction enhanced miR-338-3p expression and reduced CyclinD1 expression in HBx-expressing cells, supporting that HBx is necessary for cyclinD1 upregulation through miR-338-3p.

The miR*-*338 gene is located on chromosome 17q25 and produces two mature forms (miR*-*338*-*3p and miR*-*338*-*5p). Our data showed that miR-338-3p expression is down-regulated in inducing tumor formation HBx-expressing cells compared with normal hepatocyte cell line LO2 and QSG7701, similar to the results found in another HCC cell line HepG2.2.15 cells [29]. Moreover, another study reported that down-regulated miR*-*338 expression, and miR-338-3p in particular, was frequently found in HCC tissues [30], which peripherally supports our data that miR-338-3p is associated with HCC formation. The miR-338 gene is located within the intron 8 region of the apoptosis -associated tyrosine kinase (AATK) gene [31]. Interestingly, the survivin gene, a new inhibitor of apoptosis protein family, is also located on chromosome 17q25 [32]. Overexpression of survivin gene was found in a wide variety of tumor and transformed cells, including liver cancer [32]–[34] and cells in chronic HBV infected livers that are deemed close to transformation to tumor cells [32], [35], suggesting that miR-338-3p may play an important role in liver cancer formation due to its location in the fragile site locus associated with liver cancer tumorigenesis. Currently, there are few studies on miR-338-3p, although it was reported that COXIV and SMO could be regulated by miR-338-3p [36]–[37]. SMO, a transmembrane protein, has a switch function in Sonic hedgehog (Hh) signaling pathway; the classic Hh signaling pathway has been associated with tumorigenesis in the literature [38]–[39], further implicating a close correlation between miR-338-3p and tumor development. The focus of our study is on CyclinD1, a novel target of miR-338-3p. G1/S-specific CyclinD1 is a protein in the highly conserved Cyclin family and functions at the transition between the G1 and S cell cycle phases where it is a key signaling protein for G1 cell proliferation [40]. CyclinD1 overexpression leads to a remarkable reduction in the lag time between the G1/S phase cell cycle transition as well as promotion of the cell cycle progression rate, eventually leading to uncontrolled cell proliferation and tumor formation. In contrast, CyclinD1 inhibition in KM20 cells by effective siRNA treatment leads to cell cycle arrest and cell growth inhibition [41]. Therefore, CyclinD1 can be considered as an oncogene [42]–[43]. Previous studies have suggested a link between HBx and CyclinD1, where CyclinD1 is shown to be up-regulated by HBx; in these studies, the process is independent of extracellular mitotic signals [44] or is mediated by the NF-κB2(p52)/BCL-3 complex [45]. However, our findings have revealed a new process to explain how HBx can up-regulate CyclinD1, and that mechanism is by down-regulating miR-338-3p. Therefore, HBx, especially the HBx-deletion mutant HBx-d382, is involved in regulating CyclinD1 expression through an HBx-mediated miR-338-3p down-regulation mechanism, suggesting that miR-338-3p plays a tumor suppressor role in the development of HBx- and HBx-d382 deletion-mutant–mediated HCC.

The effects of HBx on cell cycle progression are potentially complicated. Most studies found that HBx stimulated cell cycle progression that accelerated transit through checkpoint controls at G0/G1 [44], [46]–[47], which is consistent with our studies. However, several other studies show that HBx actually inhibited cell proliferation by using Hepa1–6 (mouse HCC), HepG2 (human HCC) [48], or hepatocytes isolated from HBx-expressing mice [49]. One possible reason for the contradictory results may be the use of different cell lines with different differentiation statuses and different genetic backgrounds. Another possibility is that the HCC tumor cells may modify the biological activity of HBx, which is something we tried to address in our present study using normal hepatocytes. Yet another possibility is that p53 levels may influence HBx function, as p53 is known interact with HBx, and the normal physiological level of p53 displays anti-apoptotic activity, whereas a high level of p53 displays an adverse result [50]–[51].

The recent studies on HBV-related HCC found that genetic heterogeneity of the HBx gene is prevalent in liver cancer tissue. For example, wild-type HBx and mutant HBx can coexist in the same tumor [10]. The major mechanism underlying the creation of HBx deletion mutants is loss of C-terminal fragments of different sizes; this is a dominant phenotype that accounts for almost 100% of the HBx present in the integrated HBV DNA [8], [10], [52]. The HBx protein functional domains are divided into the regulatory region and the trans-activation region, where the regulatory region is located near the N-terminal end (1∼50 aa) and the trans-activation region is located near the carboxyl terminus (51∼154 aa) end. The 1∼20 aa in the regulatory region is responsible for inhibiting the activity of the trans-activation region [53]. Therefore, a point mutation or deletion mutation occurring at almost any region in the HBx gene could affect its trans-activation function. Since the deleted region of the HBx-d382 (nt 382–400 deletion) mutant is located near the C-terminal trans-activation region and is also close to where the trans-activation domain associates with mitochondria in HBV-infected cells (the first l32∼139 amino acids), the deleted region is necessary for HBx trans-activation activity as well as its known association with mitochondria. Therefore, the HBx-d382 mutant has a close correlation with the process of HBx gene replication and transcription, which are involved in the viral-host interaction, as well as the apoptosis machinery located in the mitochodria. While the loss of C-terminal expression in HBx-d382 mutant attenuates the effect of wild-type HBx on cell proliferation, the expressed truncated HBx protein has gained the ability to promote the malignant transformation of cells. In addition to the role described here, the deleted region in the HBx-d382 mutant is also known to be involved in the p53-binding region of the HBx gene (102∼136 aa). Direct binding of HBx to human tumor suppressor p53 has been reported to inhibit p53-stimulated transcription; additionally, the p53 and HBx interaction also reduced the HBx-mediated trans-activation [54]. Therefore, loss of the p53 binding site in HBx mutants can affect the tumor-suppression ability of p53 and further promote tumor formation. Taken together, these results collectively suggest that multiple HBx gene mutations found in HCC, including HBx-d382, may promote the development of HBx-mediated liver cancer.

In conclusion, our study revealed that the HBx-d382 mutant has an inhibitory effect on miR-338-3p expression that is associated with HBx-d382-mediated promotion of liver cell proliferation. The finding that HBx-d382 attenuated the miR-338-3p-mediated inhibition of CyclinD1 expression may provide insight into HBx-mediated tumorigenesis and a new direction for further investigation into HBx function and therapeutic development.

## Supporting Information

Figure S1 **miR-338-3p expression in normal hepatocytes of LO2 and QSG7701 cells compared with HBx-expressing cells by real-time PCR.** (A) Relative expression of miR-338-3p in engineered LO2 cells. 1: LO2; 2: LO2/pcDNA3.0; 3: LO2/HBx; 4: LO2/HBx-d382. (B) miR-338-3p expression in QSG7701 cells transfected with HBx using real-time PCR. 1: QSG7701; 2: QSG/pcDNA; 3: QSG/HBx; 4: QSG/HBx-d382 (*p>0.05, **p<0.001).
(TIF)

Figure S2 **Cell cycle analysis of control LO2/pcDNA3.0 cells.** Histograms of average of G1/S phase populations in LO2/pcDNA3.0 cells after transfection with miR-338-3p mimics or inhibitor (*P<0.001, **P<0.01).
(TIF)

Figure S3 **miR-338-3p and CyclinD1 expression after knocking-down HBx in HBx-expressing cells.** (A–B) HBx mRNA and protein expression levels after transfection with HBx siRNA compared with control RNA in LO2/HBx and LO2/HBx-d382 cells (*P<0.001). (C) Relative expression of miR-338-8p using the 2^−ΔΔCT^ method of qRT-PCR after altering HBx in LO2/HBx and LO2/HBx-d382 cells (*P = 0.013,**P = 0.008). (D) CyclinD1 levels in HBx-expressing cells after transfection of the HBx siRNA or negative control (***P<0.001). Data are shown as mean ±SD of 3 separate experiments.
(TIF)
